# Chest CT Findings and Differential Diagnosis of *Mycoplasma pneumoniae* Pneumonia and *Mycoplasma pneumoniae* Combined with Streptococcal Pneumonia in Children

**DOI:** 10.1155/2021/8085530

**Published:** 2021-06-14

**Authors:** Jing Wang, Chen Xia, Ashutosh Sharma, Gurjot Singh Gaba, Mohammad Shabaz

**Affiliations:** ^1^Department of Infectious Diseases, Children's Hospital of Nanjing Medical University, Nanjing, Jiangsu 210008, China; ^2^Institute of Computer Technology and Information Security, Southern Federal University, Rostov-on-Don, Russia; ^3^School of Electronics and Electrical Engineering, Lovely Professional University, Phagwara 144411, India; ^4^Arba Minch University, Arba Minch, Ethiopia

## Abstract

**Background:**

In this day and age, 17% of children less than 5 years of age died of pneumonia; it is the common cause of children death. It is one of the main children respiratory infectious diseases, i.e., mycoplasma pneumonia (MP). The imaging examination can be adopted to quickly observe the morphology and scope of the pulmonary lesions and know the effect of disease treatment and subsequent changes in the disease in order to provide a basis for treatment. Therefore, the most commonly applied technology for detecting pneumonia in children is imaging technology, including chest X-ray and CT.

**Objectives:**

The main objective of the work is to investigate the chest computed tomography (CT) findings of children patients with *Mycoplasma pneumoniae* pneumonia (MPP) and MP combined with streptococcal pneumonia (SP). The mixed infection of MP and SP is very common clinically, and the diagnosis of this type of mixed pneumonia is a critical research topic faced by pediatric respiratory physicians. The comparison is done on the incidence of bronchial and pulmonary interstitial lesions, the degree of lymph node enlargement, the volume and depth of pleural effusion, and the location and morphology of the pulmonary lesions in the chest CT images of children patients from the two groups.

**Methods:**

There were comparisons on the incidence of bronchial and pulmonary interstitial lesions, the degree of lymph node enlargement, the volume and depth of pleural effusion, and the location and morphology of the pulmonary lesions in the chest CT images of children patients from the two groups. All the experiments are done in the MATLAB.

**Results:**

The results showed that the proportions of reticular shadow, ground glass shadow, bronchial inflation phase, tube wall thickening, and vascular bundle thickening on the CT images of children patients from the MPP group were dramatically higher than those of the MP + SP group (*P* < 0.05). The maximum transverse diameter of enlarged lymph node in children patients from the MPP group was obviously larger than the diameter of the MP + SP group (*P* < 0.05). The number of children patients with pleural effusion was 22 in the MP + SP group, which was greatly higher than the MPP group (*P* < 0.05).

**Conclusion:**

In conclusion, the chest CT images of children patients from the MPP group were mainly pulmonary interstitial changes. Furthermore, the alveolar inflammation could be observed on the CT images shown when children patients were combined with SP infection. The more obvious manifestations were that the flaky shadows appeared in the lungs, the pleural effusion became thicker, and the transverse diameters of enlarged lymph nodes were bigger.

## 1. Introduction

Childhood pneumonia is the main cause of death for children under the age of 5 years, and SP is the most common type of pneumonia from the 20^th^ day of birth to the entire childhood. The MP infection rate in children that are older than 5 years old is more than 50% [1]. The mixed infection of MP and SP is very common clinically, and the diagnosis of this type of mixed pneumonia is a critical research topic faced by pediatric respiratory physicians. Accurate imaging diagnosis can help clinicians to treat the disease in time and use drugs rationally, so as to avoid delay in the conditions of patients.

Nowadays, 17% of children less than 5 years of age died of pneumonia; it is the common cause of children death [2, 3]. It is one of the main children respiratory infectious diseases, that is, mycoplasma pneumonia. In the initial age, there may or may not be clinical symptoms which cause the lesions outside the respiratory system. Several days are required for the completion of the serologic diagnosis for making decision of initial medication which is critical for the community-acquired pneumonia treatment [3]. The images for childhood pneumonia and the fight against pneumonia are shown in Figure 1.

Pneumonia is the most frequent disease and its main causes are pathogen infection and body allergic reactions. In the past 3 years, MPP has become a common pneumonia in children and adolescents, accounting for 10%–40% of community-acquired pneumonia, and its infection rate is 10%–20% [4, 5]. Compared with simple MP, combined SP is more likely to cause severe pneumonia. It can damage the pulmonary tissue and seriously endanger the health of children. Clinical studies have confirmed that mixed-infected children with pneumonia have a longer course and are more likely to develop pulmonary lesions and pleural effusion. Among them, SP is the most common [6] and it is gradually being paid attention to in clinic. Thus, effective identification of MP infection and mixed infection of MP and streptococcus has vital reference significance for the treatment of childhood pneumonia. The imaging examination can be adopted to quickly observe the morphology and scope of the pulmonary lesions and know the effect of disease treatment and subsequent changes in the disease in order to provide a basis for treatment. Therefore, the most commonly applied technology for detecting pneumonia in children is imaging technology, including chest X-ray and CT.

The multislice spiral CT method is used with a scanning layer, and there are different conditions for scanning. Regular chest CT scans of children are done in calm breathing state. The underwent breathless scanning is held by the older children. The MP antibody is detected by the passive agglutination method (MP-IgM) with patient's serum twice every 10 or 14 days [7]. The two experienced radiologists assessed the CT imaging and retrospectively diagnosed the diseases including the lesion characteristics and lesions involving lobes. The ground glass opacity (GGO), the consolidation opacity, and the mass opacity are included by the lesion types. Peribronchovascular nodules are presented in the bronchovascular bundle, and mildly increased attenuation without obscuration of the underlying vasculature is known as GGO [8, 9]. There are three types of nodules:

1. Centrilobular nodules in the centrilobular location
2. Peribronchovascular nodules in the bronchovascular bundles
3. Granulomas

Studies have shown that interstitial changes are the pathological basis of MPP [10]. It is the first to damage the body's terminal and respiratory bronchiolar epithelial cells, so as to cause the parabronchial tissues to infiltrate into the interlobular septum, thereby resulting in thickening of the interlobular septum and edema of the bronchiole wall. The lesions are mainly concentrated in the small and medium airways [11]. The cuffing signs and thickening of the bronchial wall can be observed in the thin-layer CT images of the chest, showing ring sign, orbit sign, and thickening of the bronchial vascular bundle [12]. If the condition is mild, the interlobular space will be thickened, and a small part of the pulmonary tissues will be also thickened. However, most will become asymmetric and irregular high-density small shadows. At this time, the lesions will merge with each other. The invasion function of bacterial capsule is the main therapeutic factor of SP. Invasion of tissues first causes edema of the alveolar wall, and then, white blood cells and red blood cells exudate. At this time, the alveoli are quickly and directly invaded by bacteria. The bacteria can even invade directly, causing symptoms such as congestion and edema in the pulmonary lobes.

Many researchers have worked on differential diagnosis of *Mycoplasma pneumoniae* pneumonia and *Mycoplasma pneumoniae* combined with streptococcal pneumonia in children for many years. The scientific basis for clinical diagnosis and severity assessment are provided for the improvement of comprehension of the imaging findings for the children chest imaging discussion. In the pediatric department, 126 cases of children are analyzed [13]. With chest computed tomography, this paper aims to clarify the abnormalities pattern with *Mycoplasma pneumoniae* pneumonia, and *M. pneumoniae* pneumonia from *Streptococcus pneumoniae* pneumonia is distinguished through the radiographic findings [14]. The CT case of different cases is performed by the retrospective review. The bilateral bronchial wall thickening or centrilobular nodules were seen in the patients. In the same patients, CT findings between early stage and progressed stage are compared and in the progressed stage, early stage radiographic features were not clearly observed. The wall thickening and centrilobular nodules in the CT outcomes are found by the *M. pneumoniae* pneumonia diagnosis. From the recent publications, the comprehensive radiological literature review is provided on ongoing radiological investigation of the imaging features of the chest ultrasound (US), radiographs (CXR), and computed tomography (CT) examinations. The evaluation and analysis of multimodality imaging outcomes are done [15]. In many patients, the different tests like chest US, CXR, and CT were performed. The glenohumeral instability of patient's MRI is analyzed, and torn labrum diagnosis is determined which can be confirmed by the surgical exploration [16]. The correct labral tear diagnoses are 80% obtained after the analysis. A clinical, radiological, and histological entity is organizing pneumonia which is classified as interstitial lung disease [17]. The new understandings of the clinical and histological presentation are summarized in this work, and the most relevant CT features are reviewed. The author in this paper details many complications like pneumonia commonly accompanied by emphysema. The usual disease progression is changed by the destroyed airspaces [18]. Various cases of common comorbidities are demonstrated by the authors with unusual radiographic findings in emphysema patients. The proper management of emphysema patients is commonly diagnosed by the various emphysema findings. In this paper, the author details the radiographic findings which are nonspecific in mycoplasma pneumonia [19]. A single lobe is confined by the focal reticulonodular opacification which is radiographic pattern and closely associated with the mycoplasma infection. The mycoplasma pneumonia diagnosis is considered when bilateral reticulonodular opacification is seen. Due to confluent interstitial shadows, transient pseudoconsolidations are seen often. For the mycoplasma pneumonia diagnosis, radiographic findings are not sufficient. By combining the clinical findings, diagnosis accuracy is increased. The author describes the radiological features in adult patients with H1N1 influenza pneumonia [20]. During the epidemic of H1N1 influenza infection, descriptive study of retrospective data is performed. By RT-PCR, H1N1 influenza virus infection is confirmed by the 209 adult patients. The opacities were mainly bilateral, basal, and midzonal in CXR and peripheral in CT. In the H1N1 pneumonia, the predominant radiological pattern is bilateral and alveolar consolidation. To maximise iodine detection, preprocessing is done by the author in this paper for chest imaging in acute and chronic embolic diseases demonstration [21]. The work aims to set out the physical basis for the technology and postprocessing protocols used and to present future developments.

The literature lacks the investigation of chest computed tomography (CT) findings of children patients with *Mycoplasma pneumoniae* pneumonia (MPP) and MP combined with streptococcal pneumonia (SP), which is very important. For the differential diagnosis references and treatment of MPP in clinic, reference is required. Clinically, the MP and SP mixed infection is very common, and the mixed pneumonia diagnosis is a critical research topic faced by pediatric respiratory physicians. In this paper, the main contribution of the work is to investigate the chest computed tomography (CT) findings of children patients with *Mycoplasma pneumoniae* pneumonia (MPP) and MP combined with streptococcal pneumonia (SP). In this study, 80 children patients with pneumonia were selected and were admitted to the Department of Respiratory Medicine of Indira Gandhi Medical Hospital from June 2019 to June 2020. Besides, 40 cases with MPP and 40 cases with MP combined with SP were enrolled into a MPP group and a MP + SP group in turn based on the results of serum MP-IgM detection and streptococcal blood culture. There were comparisons on the incidence of bronchial and pulmonary interstitial lesions, the degree of lymph node enlargement, the volume and depth of pleural effusion, and the location and morphology of the pulmonary lesions in the chest CT images of children patients from the two groups.

## 2. Materials and Methods

### 2.1. Clinical Research Objects

From June 2019 to June 2020, 80 children patients admitted to the Department of Respiratory Medicine of Indira Gandhi Medical Hospital for one year were selected as the research objects, who suffered from MMP and MP combined with SP confirmed by blood culture and serological examinations in turn. Among them, there were 40 cases in the MPP group, including 19 boys and 21 girls. Besides, they were 3–12 years old, with an average age of 7.50 ± 2.66 years [22–24]. There were also 40 cases in the MP + SP group (22 boys and 18 girls), with the age of 5–14 years (average age of 8.78 + 2.99 years). The differences in gender and age of the two groups were not statistically obvious (*P* > 0.05). All children patients underwent chest CT detections before receiving antibiotic treatment.

### 2.2. Operating Equipment and Methods

The children patients from the MPP group and the MP + SP group were given with chest CT scanning before treatment. The multislice spiral CT machine was adopted in this experiment [25]. What's more, they were asked to maintain breath-holding during the examination. The scanning range included chest cavity to lung base, with the adjustment of related parameters, and the corresponding data were uploaded to the workstation after scanning.

### 2.3. Observation Indicators

The 3 experienced imaging doctors examined all the research objects in this study and observed the CT images together in terms of the signs of bronchial and pulmonary interstitial lesions, the transverse diameter of lymph nodes and other specific manifestations, and the incidence and depth of pleural effusion. Then, the location and morphology of lesions in children patients from the two groups were analyzed based on the above observation indicators. According to these symptoms in children with pneumonia, the corresponding lesions might be judged [26, 27]. The lesion distribution presented on the CT images could be classified into consolidation, ground glass shadow, and reticular shadow on the basis of imaging density and divided according to lung lobes (anatomical unit) into left and right sides, and upper and lower lobes.

### 2.4. Statistical Methods

The measurement data were represented by mean ± standard deviation ($\bar{x}$ ± *s*), and the disordered classification data were expressed as percentage (%). SPSS 20.0 software was employed to analyze the difference between the two groups [28]. Above all, *P* > 0.05 meant that the difference was not statistically substantial, and *P* < 0.05 indicated there was a statistically marked difference.

### 2.5. Clinical Features of Mycoplasma Infection

For mycoplasma pneumonia, humans are the only known reservoir. It is the tiny organism which is less than 350 *μ*m and not visible at light microscopy [5]. This infection is spread by direct contact for the period of 1-2 weeks. It is an important cause of community-acquired respiratory infections in school-age children. Mycoplasma pneumonia illness is gradual, and its symptoms are nonspecific. The illness may begin in the upper respiratory tract and is often accompanied by low-grade fever, headache, and myalgias [29–32]. The rales, rhonchi, and decreased breath sounds are the different clinical signs included in the lungs mycoplasma infection. Usually the white blood cell count is in normal range. The respiratory symptoms precede the nonrespiratory manifestations in most of the cases, but there is little effect of pulmonary disease on subsequent neurologic disease [33].

## 3. Results and Discussion

### 3.1. Children with Bronchial and Interstitial Lung Disease from the Two Groups

The chest CT findings of bronchial and pulmonary interstitial lesions in children patients from the MPP group and MP + SP group were observed and compared, and the comparison results are shown in Table 1 and graphically shown in Figure 2. The CT images of children patients from the MPP group showed reticular shadows, ground glass shadows, reticular shadows, bronchial inflation phase, tube wall thickening, and vascular bundle thickening, and the appearance proportion of the above in the MPP group was higher obviously than that of the MP + SP group (*P*=0.03 and *P* < 0.05) [34]. Besides, Figure 3 indicates the specific signs of chest CT in one child patient from the MPP group (the image of this patient was typical). The proportions of cases with bronchopulmonary emphysema and bronchial inflation phase from the two groups were compared, with no statistically obvious difference (*P*=0.94 and *P* > 0.05).

### 3.2. Children with Pleural Effusion and Lymph Node Enlargement from the Two Groups

The largest transverse diameter of enlarged lymph nodes in the MPP group and the MP + SP group was 7.23 ± 2.38 mm and 9.68 ± 2.95 mm, respectively. It was found that the transverse diameter of enlarged lymph nodes in children patients from the MP + SP group was greatly larger than that of the MPP group (*P*=0.04 and *P* < 0.05) (Table 2). The depth of pleural effusion in children patients from the MPP group was 3.35 ± 2.23 mm, while the depth of the MP + SP group was 12.75 ± 11.36 mm [35, 36]. Thus, the depth of pleural effusion in children patients from the MP + SP group rose hugely in contrast to the depth of the MPP group (*P*=0.009 and *P* < 0.05).  Figure 4 shows that the incidence of pleural effusion in children patients from the MPP group (22%) reduced steeply in contrast to the incidence of the MP + SP group (55%) (*P*=0.031 and *P* < 0.05).

### 3.3. The Pathogenic Sites in the Lungs of the Sick Children

There was a comparison of the pathogenic sites of children patients from the MPP group and MP + SP group (*P* > 0.05), and the results are presented in Tables 3 and 4 and graphically shown in Figures 5 and 6 for better analysis and visualization.

### 3.4. Morphology of Pulmonary Lesions in Sick Children

In the MPP group, 33 cases had fan-shaped thin slice shadows in the lungs, and the incidence was 83%. Besides, there were 7 cases with fan-shaped thin slice shadows in the MP + SP group (18%). Thus, the above was statistically different (*P* < 0.05). As for irregular pulmonary consolidation, there were 36 in the MP + SP group (90%) and 9 in the MPP group (23%), and the difference was statistically substantial (*P* < 0.05) (Figure 7).

The results of this study revealed that the proportion of reticular shadow, ground glass shadow, bronchial inflation phase, tube wall thickening, and vascular bundle thickening in chest CT images of the MPP group was markedly higher than that of the MP + SP group. The damage of MPP was most representative in the terminal and respiratory bronchiole epithelium, so the accumulation and infiltration of mononuclear lymphocytes will occur in some tissues clinically, and eventually the symptom of bronchopulmonary emphysema will appear. Therefore, thickening of the bronchial wall and the bronchial vascular bundle could be discovered on the chest CT images. With the progression of the disease, the surrounding tissues of the bronchiole would be infiltrated by inflammation again, so that the interlobular septa were thickened [37–39]. The alveolar cavity was the main site of SP inflammation, leading to the symptoms of pulmonary congestion and edema.

## 4. Discussion

The inflammatory response of MP combined with SP is more severe than that of MPP alone, and it is manifested as a more substantial local inflammatory exudation rate and less air bubbles in the alveolar cavity. On the CT images, the translucency of the lung field was reduced [40–42]. However, a large area of dense shadows in the lungs could be observed on the CT images when a large amount of inflammatory exudation led to the loss of air in the alveoli, which could block the pulmonary interstitial changes caused by MPP [43]. Therefore, the proportion of ground glass shadow and reticular shadow in children patients from the MP + SP group decreased sharply. Studies have pointed out that hilar lymph node enlargement has occurred in about 1/5 of patients with pneumonia, most of which have been unilateral. Lymph node enlargement behind the anterior tracheal vena cava was observed in all children patients in this study, which was basically the same as the research results of relevant literature. In addition, the maximum transverse diameter of lymph node enlargement in children patients from the MPP group (7.23 ± 2.38 mm) dropped hugely compared with the MP + SP group (9.68 ± 2.95 mm). It indicated that children patients with obvious lymph node enlargement in the actual clinical setting had the possibility of mixed infection; for example, the maximum transverse diameter was more than 0.9 cm.

In this study, the incidence of pleural effusion in children patients from the MPP group was 22%, while the incidence of pleural effusion in the MP + SP group was 55%. Thus, the above incidence of the MP + SP group was dramatically higher than that of the MPP group, which was mainly caused by the inflammatory exudation after MP infection and the induced pleural response [44–46]. Inflammation can further enhance the permeability of the local capillary wall. At this time, the inflammatory exudate increases, thus making the pleural effusion obviously more. For all the children patients with pneumonia with relatively more pleural effusion, the possibility of suffering from MP combined with SP could not be excluded.

From the perspective of the pathogenesis of MPP and SP, there is little difference in the sites of the two types of pneumonia. It was consistent with the research of left and right pulmonary lesions in this study. Left lung lesions were slightly greater than right lung lesions, but there was no difference between the two types of pneumonia.

In this study, the irregular pulmonary consolidation shadows appeared in the CT images of 36 children patients from the MP + SP group, with an incidence of 90%, which was markedly higher than the incidence of the MPP group. There were consolidation shadows with irregular shapes after the onset of lesions, and this was because of the result of lesion fusion due to the inflammation of alveoli. It was also in line with the pathologic findings of MP combined with SP.

## 5. Conclusion

Pneumonia is the most frequent disease in children, and its main causes are pathogen infection and body allergic reactions. In the past 3 years, MPP has become a common pneumonia in children and adolescents, accounting for 10%–40% of community-acquired pneumonia, and its infection rate is 10%–20%. For the sake of medical ethics, the differences in the two types of pneumonia were observed on the basis of CT detection. However, there is a lack of comparison of the chest X-ray examinations of children patients from the two groups. The 3 experienced imaging doctors examined all the research objects in this study and observed the CT images together in terms of the signs of bronchial and pulmonary interstitial lesions, the transverse diameter of lymph nodes and other specific manifestations, and the incidence and depth of pleural effusion. Then, the location and morphology of lesions in children patients from the two groups were analyzed based on the above observation indicators. It is planned to carry out further comparison of the differential diagnosis between the two groups by chest X-ray examination, which may be more convincing and is better to expand the application of chest X-ray in the treatment of MPP and SP. The irregular pulmonary consolidation shadows appeared in the CT images of 36 children patients from the MP + SP group, with an incidence of 90%, which was markedly higher than the incidence of the MPP group; the alveolar inflammation could be observed on the CT images shown when children patients were combined with SP infection. The more obvious manifestations were that the flaky shadows appeared in the lungs, the pleural effusion became thicker, and the transverse diameters of enlarged lymph nodes were bigger. There were consolidation shadows with irregular shapes after the onset of lesions, and this was because of the result of lesion fusion due to the inflammation of alveoli. It was also in line with the pathologic findings of MP combined with SP. The investigation of the emerging COVID-19 pneumonia's imaging features on chest ultrasound (US) and computed tomography (CT) examinations can be focused on in the future research.

## Figures and Tables

**Figure 1:** (a) Childhood pneumonia. (b) Fight against pneumonia.

**Figure 2:** Chest CT findings and infection rate of bronchial and pulmonary interstitial lesions.

**Figure 3:** Chest CT image of one child patient from the MPP group.

**Figure 4:** The incidence of pleural effusion in children patients from the two groups.

**Figure 5:** Left lung lesions of children patients from the two groups.

**Figure 6:** Right lung lesion sites of children patients from the two groups.

**Figure 7:** The incidence of two types of pulmonary lesions in children patients from the two groups.

**Table 1:** Chest CT findings and infection rate of bronchial and pulmonary interstitial lesions in children patients from the MPP group and MP + SP group (%).

Chest CT findings	MPP group (*n* = 40)		MP + SP group (*n* = 40)	
	Number of cases	Infection rate (%)	Number of cases	Infection rate (%)
Bronchopulmonary emphysema	8	15	10	25
Reticular shadow	34	80	12	30
Ground glass shadow	24	60	7	18
Bronchial inflation phase	37	93	32	80
Tube wall thickening	38	95	20	50
Vascular bundle thickening	32	70	13	33

**Table 2:** Comparison of the depth of pleural effusion and the maximum transverse diameter of lymph nodes in children patients from both groups ($\bar{x}$ ± *s*).

Group	Depth of pleural effusion	Maximum transverse diameter of lymph nodes
MPP group (*n* = 40)	3.35 ± 2.23	7.23 ± 2.38
MP + SP group (*n* = 40)	12.75 ± 11.36	9.68 ± 2.95
*P* value	<0.05	<0.05

**Table 3:** Comparison of the left lung lesions of children patients from the two groups.

Group	Number of cases	Left lung			
		Upper lobe		Lower lobe	
		Number of cases	%	Number of cases	%
MPP group	40	20	50	14	35
MP + SP group	40	15	38	17	43
*P* value		>0.05			

**Table 4:** Comparison of the right lung lesion sites of children patients from the two groups.

Group	Number of cases	Right lung					
		Upper lobe		Middle lobe		Upper lobe	
		Number of cases	%	Number of cases	%	Number of cases	%
MPP group	40	10	25	14	35	11	28
MP + SP group	40	13	33	12	30	15	38
*P* value		>0.05					

## Data Availability

The data are available upon request to the corresponding author.
